The article "Metagenome-assembled genomes infer potential microbial metabolism in alkaline sulphidic tailings" was retracted in 2024. Reasons: no approval from the institution; concerns about the data.

# Metagenome-assembled genomes infer potential microbial metabolism in alkaline sulphidic tailings

**DOI:** 10.1186/s40793-021-00380-3

**Published:** 2021-04-29

**Authors:** Wenjun Li, Xiaofang Li

**Affiliations:** 1 Hebei Key Laboratory of Soil Ecology, Key Laboratory for Agricultural Water Resource, Center for Agricultural Resources Research, Institute of Genetics and Developmental Biology, Chinese Academy of Sciences, Shijiazhuang, 050021 China; 2 University of Chinese Academy of Sciences, Beijing, 100049 China

**Keywords:** Sulphidic tailings, Metagenomics, Binning, Community genomics, Sulphide oxidation

## Abstract

**Background:**

Mine tailings are hostile environment. It has been well documented that several microbes can inhabit such environment, and metagenomic reconstruction has successfully pinpointed their activities and community structure in acidic tailings environments. We still know little about the microbial metabolic capacities of alkaline sulphidic environment where microbial processes are critically important for the revegetation. Microbial communities therein may not only provide soil functions, but also ameliorate the environment stresses for plants’ survival.

**Results:**

In this study, we detected a considerable amount of viable bacterial and archaeal cells using fluorescent in situ hybridization in alkaline sulphidic tailings from Mt Isa, Queensland. By taking advantage of high-throughput sequencing and up-to-date metagenomic binning technology, we reconstructed the microbial community structure and potential coupled iron and nitrogen metabolism pathways in the tailings. Assembly of 10 metagenome-assembled genomes (MAGs), with 5 nearly complete, was achieved. From this, detailed insights into the community metabolic capabilities was derived. Dominant microbial species were seen to possess powerful resistance systems for osmotic, metal and oxidative stresses. Additionally, these community members had metabolic capabilities for sulphide oxidation, for causing increased salinity and metal release, and for leading to N depletion.

**Conclusions:**

Here our results show that a considerable amount of microbial cells inhabit the mine tailings, who possess a variety of genes for stress response. Metabolic reconstruction infers that the microbial consortia may actively accelerate the sulphide weathering and N depletion therein.

## Introduction

Mine tailings are milled residue wastes of ore processing. Those of metal mines, typically Pb/Zn/Cu/Ni, always contain abundant sulphides that are mostly pyrite based, e.g. FeS_2_. Due to the high reactivity of sulphides, high levels of metals and salinity can be generated by the coupled weathering of sulphide and carbonate wastes [1]. This makes mine tailings a rather hostile environment to microbes, while still a considerable amount cells, though with a relatively low diversity compared with normal soils, had been detected therein [1]. The contribution of microbial activities to the weathering of sulphides has long been recognized in mine tailings. At the acid mine drainage (AMD) site of Iron Mountain, Calif., *Thiobacillus ferrooxidans* and *Leptospirillum ferrooxidans* were found to be dominant in the community and contribute to the generation of AMD [2]. In a copper bioleaching heap, sulfurophilic and iron-ophilic acidophilic bacteria were found to actively colonize the mineral surface [3]. These microbes show adaptability to extremely acidic environment and play an important role in the sustainability of this system. With the advent of the modern molecular tools, community genomics of microbial consortia in acid mine environments has been well explored [4, 5], while that of alkaline mine tailings has not been extensively studied. Alkaline mine environment is normally subjected to revegetation which requires the establishment of soil function including microbial diversity [6].

Microbial community networks related to sulphide weathering in neutralized tailings have been determined [7, 8], yet these studies are based on mainly 16S rRNA gene detection and then possible functions of the community members are inferred from physiological information of known related pure cultures. This approach is useful but is highly limited and speculative with regard to approximating the community metabolic capabilities related to the in situ elemental cycling and adaptation strategies. In contrast, metagenome-based analyses enable reconstruction of nearly complete genomes of microbial community members. Such analyses provides detailed insights of metabolic capabilities and enables estimating the possible contributions of populations to the community processes [5]. Metagenomic approaches have been successfully used to resolve the microbial biogeochemical potential in saline sea water [9, 10], and to reconstruct microbial metabolism in AMD. It is found that acidophilic bacteria community in AMD has a microbial diversity higher than expected [11, 12]. Recently, draft genomes acquired through metagenomics have been used to understand the bacterial colonization of the infant gut [13] and microbial systems in hypersaline lakes [14].

In this study, we analyzed metagenomes of alkaline sulphidic tailings from a tailings storage facility of northwest Queensland. Microbial metabolic capabilities for stress resistance and elemental cycling were implied through the annotation of 10 metagenome-assembled genomes (MAGs) from the tailings metagenomes. The results may provide further understanding on biogeochemistry of alkaline sulphidic tailings and valuable inference for tailings revegetation practice.

## Materials and methods

### Sampling

Sampling sites and methods have been described in our previous studies [15, 16]. Briefly, base metal mine tailings were sampled from a storage facility Mt Isa, northwest Queensland. The microbial community structure based on 16S rRNA gene sequencing related to revegetation has been determined and described elsewhere. The tailings mainly comprise of quartz, dolomite, pyrite, gypsum and kaolinite, and contain approximately 1300, 1800 and 2900 mg/kg of residue Cu, Pb and Zn, respectively. The 16S-based amplicon sequencing reveals that the dominant microbial species in the tailings include *Rubrobacter* spp. of the *Actinobacteria*, *Truepera* spp. of the *Deinococcus-Thermus,* and *Thioalkalivibrio* spp. and *Thiobacillus* spp. of the *Proteobacteria*. No substantial changes were detected of the microbial community structure in summer and in winter [6], and dominant species changed little in spite of significant increases in diversity detected along with the revegetation efforts [15].

### Fluorescent in situ hybridization (FISH)

Cells from the tailings samples were firstly enriched by a sucrose density centrifugation [17], followed by the standard FISH procedure for soil with minor modifications [18, 19]. To obtain sufficient microbial cells from the tailings, quadruplicates with 5 g of tailings each were used for cell enrichment. Oligonucleotide probes were used for detecting bacteria (mixed EUB338) and archaea (ARCH915) [20]. The hybridized samples were observed within 24 h of performing the FISH and images were taken using a ZEISS LSM 510 META Confocal Microscope. For enumeration of microorganisms, from each sample a total of 30 confocal acquisitions were taken, and 21 quality images were used to determine the cell abundances using DAIME 1.3 [21].

### DNA extraction and sequencing

DNA extraction was done using the PowerSoil® DNA Isolation Kit (MO BIO Laboratories, Inc.), after cell enrichment using the previously described protocol [17]. A total of seven DNA samples of tailings samples were subjected to shotgun sequencing. The sequencing was done at the Institute for Molecular Bioscience, The University of Queensland, using Illumina MiSeq with paired-end 300 bp reads. The detailed sequencing method is described in our previous study [16].

### Bioinformatics

For the purpose of high quality assembly of the metagenome, the seven metagenomes were pooled together and analyzed using the flexible pipeline MetaWRAP [22] for genome-resolved metagenomic data analysis. The assembly module was used for sequence assembly. The assembly contigs obtained were all longer than 1000 bp. The workflow of MaxBin2 in MetaWRAP was used for contig encapsulation. MetaWRAP provides three assembly pipelines, namely Concoct, Metabat2 and Maxbin2, and after comparison Maxbin2 was chose for subsequent analysis [23]. Then the obtained bins were further analyzed for species annotation. Species annotation was performed in the annotate_bins module, based on the NCBI_nt and NCBI_tax databases. Taxator-tk was used for the classification of each contig, and a bin as a whole was estimated to annotate species. CheckM was used for the quality assessment of the assembled bins (MAGs; https://ecogenomics.github.io/CheckM/). For gene annotation, a cutoff E value of 10^− 6^ and an identity of 70% were used. Metawrap was run on a 42-core, 192 GB RAM server. Bins were then used for microbial metabolic pathway analysis using the online analysis platform KEGG [24].

## Results and discussion

### The environment

The tailings studied are basically neutral/alkaline in pH and of a high level of residue heavy metals, salinity and sulphidic minerals. Salinity and metal release in sulphidic tailings is mostly from the coupled weathering of sulphides and carbonates. The microbially-mediated and chemical-mediated weathering of sulphides would have both occurred in the amended and revegetated tailings [15]. The microbial processes may become as important as the chemical weathering processes in neutral/alkaline sulphidic tailings, where the redox potential of oxygen and ferric is reduced by the high pH and ferrous can be oxidized more easily with diverse electron-acceptors (e.g. nitrate) [25]. Moreover, increased nutrients supplied from the organic matter amendment and plant roots, as indicated by our previous studies, is very likely resulting in increased activities of the sulphide weathering microorganisms [6].

### Cell abundance in the tailings

Cell abundance in the tailings was enumerated using conventional FISH. We examined samples by FISH that were prepared as either sterilized raw tailings, the raw tailings or a cell enrichment obtained from the tailings by sucrose density gradient centrifugation. Strong background fluorescence was observed and direct observation of cell fluorescence was impossible for raw tailings materials. Background fluorescence is a common problem for cell enumeration in soil-like materials using FISH, and can be strong in metal tailings due to the presence of abundant uranium, lead and molybdenum minerals.

The FISH images taken on tailings samples prepared by cell enrichment were of good quality and suitable for cell enumeration (Fig. 1). The bacterial cell number in the tailings was estimated to be approximately 10^7^ cells/g tailings, assuming the cell extraction efficiency to be 10%. Bacteria made up the major component of the cells and Archaea were only scarcely detected. We did not detect any difference of the cell abundances between the tailings with and without revegetation. The bacterial and archaeal cell abundances in these tailings is close to those reported for other base metal tailings [7, 20].

**Fig. 1:** A representative FISH image (magnification, × 100) of the bacterial (green, FITC dyes) and archaeal cells (red, Cy3 dyes) detected in the tailing

### The community genomics

The analysis of 5 Gb of sequenced DNA obtained from the tailing samples resulted in 10 genomic bins belonging to eight genera (Table 1). Five of the 10 MAGs, *Rubrobacter* sp., *Truepera* sp., *Thioalkalivibrio* sp., *Acidimicrobium* sp. and *Rhodomicrobium* sp., had high completeness of > 90% and a contamination rate of 1.35–4.87%. Our previous studies based on 16S rRNA amplicon sequencing showed that these 5 genera on average accounted for > 12% of the total communities in the tailings sampled. These 5 MAGs were of high quality, which were binned with an N_50_ of 9307–32,314 bp, with the longest contigs ranging between 51,994–209,767 bp and the number of coding sequences ranging between 2963 and 4168. Five other bins were obtained of a lower quality but with a completeness > 50%. These results enabled the metabolic capacities of the communities to be determined and these capacities could be related to the tailings’ bio-weathering. All the microbial genetic features discussed here were based on the annotation of contigs with a length > 8000 bp. Restricting the analyses to large contigs would serve to minimize system errors such as those caused by sequencing and bioinformatic assembly. This metagenomic-based analysis allows a comprehensive estimation of the community metabolic networks [5]. Additionally, the sequencing depth obtained here was much greater than that of previous metagenomic studies of other tailings communities [26], which in this instance enabled good estimations of the community metabolic capabilities.

**Table 1:** General properties of the binned population genomes

Bin	Closest species	Bin size (bp)	N_50_	Longest contig (bp)	Bin completeness	GC content (%)	Number of CDS	Number of RNAs	Annotated (%)
T1	*Rubrobacter xylanophilus*	4,197,005	32,314	20,9767	94	66.1	4168	57	42
T2	*Truepera radiovictrix*	3,255,015	12,637	53,587	90	69.3	3046	35	41
T3	*Thioalkalivibrio* sp.	3,135,801	16,696	69,403	91	64.1	2923	44	47
T5		2,249,954	7700	41,708	51	65.8	1988	22	15
T10		3,250,127	1063	13,563	78	62.0	2510	41	35
T4	*Acidimicrobium ferrooxidans*	3,035,868	37,225	201,471	95	68.8	2983	49	39
T8	*Rhodomicrobium vannielii*	3,603,927	9307	51,994	94	64.0	3429	59	41
T9	*Desulfuromonas acetoxidans*	1,678,559	1063	17,628	63	38.3	1385	32	15
T17	*Thiobacillus denitrificans*	3,570,600	1305	8554	50	60.1	2903	44	21
T18	*Erythrobacter litoralis*	4,900,514	848	9004	60	64.3	3638	56	36

Key populations from the near complete MAGs, *Rubrobacter* sp., *Thioalkalivibrio* sp. and *Thiobacillus* sp., were identified to have prominent capacities for acquiring energy and stress resistance in the tailing environment (Table 2). *Rubrobacter* sp. had a wide spectrum of genes for utilizing polysaccharides and aromatic compounds, such as the *pca* [27], *sal* [28], *cat* [29] and *bpa* [27] operons. This kind of capability would be particularly important considering tailings are an oligotrophic environment [15], and in this instance, the organic amendment for revegetation in the form of woodchips would have caused an increase in content of polysaccharides and chitin [30]. However, it is worth noting that the N content of the tailings and woodchips was very low, which would have impeded the decomposition of the woodchips in the long run [31]. Our recent studies report a very slow decomposition of litter amendment in the tailings. Nonetheless, the utilization of diverse organic molecules such as polysaccharides and aromatic compounds may be a vital survival strategy for these microbes after depleting easily labile and soluble organic carbon.

**Table 2:** Genetic features detected in the binned genomes from the Mt Isa mine tailings

	Features	*Rubrobacter xylanophilus*	*Truepera radiovictrix*	*Thioalkalivibrio* sp.	*Acidimicrobium ferrooxidans*	*Rhodomicrobium vannielii*	*Desulfuromonas acetoxidans*	*Thiobacillus denitrificans*	*Erythrobacter litoralis*
Carbon metabolism	*cbb*	**√**		**√**		**√**		**√**	
	*cox*	**√**			**√**	**√**			
	*pca*	**√**							
	*sal*	**√**				**√**			
	*cat*	**√**							**√**
	FAHF	**√**			**√**	**√**			**√**
	*bph*	**√**		**√**	**√**				
	*malE*	**√**	**√**	**√**					
Sulfur metabolism	*sox*			**√**	**√**			**√**	
	Blr3520			**√**				**√**	
	*dsr*			**√**	**√**			**√**	
Nitrogen metabolism	*nos*			**√**				**√**	
	*nor*			**√**				**√**	
	*nar*	**√**		**√**	**√**			**√**	**√**
	*nir*	**√**	**√**	**√**					**√**
	*nap*								
	*nas*	**√**		**√**		**√**		**√**	
	*nrf*								
	NaT			**√**	**√**	**√**			**√**
	NiT	**√**				**√**		**√**	**√**
	*nif*				**√**				
	*urt*			**√**					
Metal resistance	*czc*	**√**	**√**	**√**	**√**	**√**		**√**	**√**
	*cus*		**√**	**√**		**√**		**√**	**√**
	*cop*	**√**	**√**	**√**	**√**	**√**	**√**	**√**	**√**
	*pco*	**√**	**√**	**√**	**√**	**√**	**√**	**√**	**√**
	*mer*	**√**		**√**	**√**	**√**		**√**	
	ACR3	**√**		**√**		**√**		**√**	**√**
	*ars*	**√**	**√**	**√**		**√**		**√**	**√**
Iron acquisition	*pit*	**√**		**√**	**√**	**√**			**√**
	SDP	**√**	**√**	**√**					
	*efu*	**√**							
Oxidative stress	GT	**√**		**√**		**√**		**√**	**√**
	Glo	**√**	**√**	**√**	**√**	**√**		**√**	**√**
	SAM			**√**		**√**			
	Fr	**√**	**√**	**√**	**√**	**√**	**√**	**√**	**√**
	NO			**√**		**√**			**√**
	SOD	**√**	**√**	**√**		**√**	**√**	**√**	**√**
Osmotic stress	*mdo*		**√**	**√**				**√**	**√**
	*bet*	**√**	**√**	**√**	**√**				**√**
	*opu*	**√**	**√**						
	SOX		**√**			**√**			
	*pro*	**√**	**√**	**√**	**√**				**√**
Mobility	*msh*			**√**				**√**	
	*flg/fli*	**√**		**√**	**√**	**√**		**√**	
	*mre*	**√**	**√**	**√**	**√**	**√**			
	*che*		**√**	**√**		**√**		**√**	

Notes: *cbb* RuBisCo genes for carbon fixation, *cox* carbon monoxide dehydrogenase genes, *pca* Protocatechuate pathway for aromatic compound catabolism, *sal* Salicylate pathway for aromatic compound catabolism, *cat* Catechol pathway for aromatic compound catabolism, *FAHF* Gentisate pathway for aromatic compound catabolism, *bph* Biphenyl pathway for aromatic compound catabolism, *mal*E Maltose ABC transporter for polysaccharides metabolism, sox Sulfur oxidation genes, *Blr3520* Conserved hypothetical genes for sulfur oxidation, *dsr* dissimilatory sulfite reductase genes, *nos* Nitrous oxide reductase genes, nor Nitric oxide reductase genes, *nar* Respiratory nitrate reductase genes, *nir* Nitrite reductase genes, *nap* periplasmic nitrate reductase genes, *nas* assimilatory nitrate reductase genes, *nrf* Cytochrome c nitrite reductase genes, *NaT* Nitrate ABC transporter genes, *NiT* Nitrite ABC transporter genes, *urt* Urea ABC transporter, *czc* Cobalt-zinc-cadmium resistance genes, *cus* Cation efflux genes, *cop* Copper resistance genes, *pco* Copper multicopper resistance genes, *mer* Mercury resistance genes, *ACR3* Arsenic resistance genes, *ars* Arsenic resistance genes, *pit* Ferric ion transporter genes, *SDP* High affinity iron transporter siderophore genes, *efu* Ferrous ion transporter genes, *GT* Glutathione S-transferase genes for oxidative resistance, *Glo* Methylglyoxal detoxification genes, *SAM* SAM-dependent mehtyltransferase genes, *Fr* Ferroxidase genes, *NO* Oxidative stress response genes, *SOD* Superoxide dismutase genes, *mdo* Glucans biosynthesis genes, *bet* Choline pathway for osmotic stress response, *opu* Choline transporter genes, *SOX* Sarcpsome oxidase genes, *pro* L-proline glycine betaine transporter genes, *msh* mannose-sensitive haemagglutinin (MSHA)-like pilus genes for cell attachment, *flg/fli* flagellar genes, *mre* rod-shape determining genes, *che* chemotaxi genes

*Thioalkalivibrio* sp., *Acidimicrobium* sp. and *Thiobacillus* sp. may have found niches within the tailings by consuming sulphides and respiring on nitrates, as inferred by the presence of sulfur-oxidizing and denitrification genes in their binned MAGs. Interestingly, *Rubrobacter* sp. and *Acidimicrobium* sp. were found to have *cox* operons for CO oxidation, inferring an ability to respire on CO. CO utilization has been documented for many microbes residing in saline environments, such as in seawater [32] and saline soils [33]. In addition, four out of the eight genera were found to contain genes for CO_2_ fixation, in the form of a minimum set of *cbbLSX* [34] (Fig. 2). The findings imply these genera can utilize atmospheric carbon sources, and this may greatly increase their survival ability in the oligotrophic tailings environment.

**Fig. 2:** A Neighbor-Joining tree showing the phylogenetics of the genes for ribulose bisphosphate carboxylase large chain of carbon fixation recovered from the binned genomes in this study. The tree was constructed using MEGA 6.06 based on the sequence alignment using the CLUSTAL method with default parameters

### Key functional genes/pathways related to the environment

The ability of microbes to cope with salinity and metal (loid) stress in the tailings was evident in the annotated MAGs. Various genes for osmotic stress resistance were detected in the MAGs of *Rubrobacter* sp., *Truepera* sp., *Thioalkalivibrio* sp., and *Acidimicrobium* sp.. These included *bet* and *pro* systems that code for the choline monooxygenase/betaine aldehyde dehydrogenase pathway [27] and for the L-proline glycine betaine ABC transport system [28], respectively. Genes coding for resistance to all the metals Zn, Cd, As, Cu and Pb were detected in all genera. Impressively, multiple copies of *czc*, encoding for Co-Zn-Cd resistance, were frequently detected in one contig (Fig. 3). All the MAGs contained both the *pco* and *cop* systems for Cu resistance, and 6 out of the 8 genera had both the ACR3 and *ars* systems for As resistance (Table 2). The high frequency of these systems emphasizes the importance of metal resistance for microbial survival in the tailings [16].

**Fig. 3:** Gene clusters for metal resistance found in the binned genomes from the Mt Isa metal mine tailings. HMT, hypothetical metal transporter gene; *czc*, cadmium-zinc-cobalt resistance gene; H, hypothetical gene; GLU, ferredoxin-dependent glutamate synthase; *ccdA*, antitoxin gene; *ars*, arsenic resistance genes; *mer*, mercury resistance genes; MDM, hypothetical metal-related genes; *tetR*, tetracycline repressor gene; *dsb*, thiol:disulfide interchange genes; *cad*, cadmium resistance genes; *cop*, copper resistance genes; *chr*, chromium resistance genes. More details can be found in the notes of Table 2

Sulphidic metal tailings are an environment where multiple stresses will occur. This includes those of oxidative damage (such as from free Fe^2+^ [32]), salinity [29], moisture content changes [34], and extremely high levels of heavy metals [33]. The Fenton reaction of intracellular Fe^2+^ by superoxide is fatal to cells [32]. We detected genes for ferroxidase (Fig. 4) and superoxide dismutases as well as genes for Fe uptake systems (e.g. Fur, *pit*) in almost all the tailings MAGs. Likely, these genes are providing these microorganisms with defenses against oxidative stress. Other protection mechanisms like methylglyoxal detoxification genes [35] and glutaredoxin genes [36] were also detected in most of the MAGs.

**Fig. 4:** A Neighbor-Joining tree showing the phylogenetics of the ferroxidase genes recovered from the binned genomes in this study. The tree was constructed using MEGA 6.06 based on the sequence alignment using the CLUSTAL method with default parameters

### Sulphide oxidation and salinity generation

KEGG annotation successfully reconstructed the metabolic capacity of sulphide oxidation and nitrogen cycling of the microbial consortia, which may be vital for the survival of the community via inter-species cooperation (Fig. 5). Two microbial pathways for sulphide oxidation, the direct contact pathway and indirect pathway [37, 38], may exist in the tailings (Fig. 5). *Thioalkalivibrio* sp., *Acidimicrobium* sp. and *Thiobacillus* sp. are well known sulfur oxidizers able to respire on sulphides [39, 40], and in this study *dsr* (organized as *dsrABCKJOPR*) and *sox* (organized as soxXYZABH) genes for sulphur oxidation were found in these three MAGs from the tailings. *Thioalkalivibrio* sp. and *Thiobacillus* sp. were both found to harbor novel conserved genes (Blr3520 genes) annotated for sulfur oxidation as well. In addition, *msh* operons encoding mannose-sensitive haemagglutinin (MSHA)-like pilus for cell attachment to substrates [41] were detected in the *Thioalkalivibrio* sp. genome. This indicated the ability of *Thioalkalivibrio* sp. to attach to pyrite surfaces for oxidation activities. Microbes can colonize and etch pyrite surfaces directly and oxidize the released sulfur, which was recently observed during ferric-catalyzed pyrite oxidation [38]. The features detected in the abovementioned genomes coincide with this model. It is thus suggested that in the oxic layer of the tailings *Thioalkalivibrio* sp., *Acidimicrobium* sp. and *Thiobacillus* sp. may colonize and oxidize sulphides particles directly, causing mineral dissolution and contributing to the elevated levels of salinity and metals in the pore water.

**Fig. 5:** A conceptual diagram depicting the microbial mediated sulphide oxidation resulting salinity and N depletion in the tailings. DMO, direct microbial oxidation; IO, inorganic oxidation; IMO, indirect microbial oxidation

Genomic features detected here also inferred an indirect oxidation of sulphides in the tailings through the coupled reactions of ferrous oxidation and nitrate reduction which may occur in an anoxic layer. Diverse ferroxidases were detected in all the MAGs (Table 2), indicating intensive microbial activities to regenerate ferric which is a strong oxidant for sulphide dissolution [38]. Additionally, a full set of denitrification genes (*nar*, *nir*, *nor*, *nos*) were detected in the *Thioalkalivibrio* sp. and *Thiobacillus* sp. MAGs. It has been determined that total nitrogen is extremely low (< 0.006%) in the tailings and most of this is in the form of microbial biomass (50–100%) [15]. There is the possibility that anaerobic microbial sulphide oxidation has occurred here with nitrate as electron acceptor. Other studies showed that pyrite minerals of nano-size were oxidized by *Thiobacillus denitrificans* with nitrate as electron acceptor [42]. Sulphides in the tailings used in this study may favor this indirect pathway due to their texture dominated by fine silt when nitrate is present. This claim about the role of nitrate in sulfide oxidation requires experimental verification in purposely designed physiological tests.

Nitrogen deficiency is a common problem in tailings limiting plant growth, and its microbial cycling has not been well studied for neutral/alkaline metal tailings [15]. Our results highlight the possibility of nitrate-depletion by microbial sulphides oxidation as well as by CO oxidation [33] in the tailings. Nitrogen fixing mechanisms in the tailings remains largely unknown. The key nitrogen fixing genes were not detected, with only *nifU* present in the *Rubrobacter* sp. and *Acidimicrobium* sp. MAGs.
